# AMPK: a therapeutic target of heart failure—not only metabolism regulation

**DOI:** 10.1042/BSR20181767

**Published:** 2019-01-03

**Authors:** Xuan Li, Jia Liu, Qingguo Lu, Di Ren, Xiaodong Sun, Thomas Rousselle, Yi Tan, Ji Li

**Affiliations:** 1 Department of Physiology and Biophysics, University of Mississippi Medical Center, Jackson, MS 39216, U.S.A.; 2 Department of Geriatrics, The First Hospital of Jilin University, Changchun 130021, China; 3 Department of Endocrinology and Metabolism, West China Hospital of Sichuan University, 37 Guoxue Lane, Chengdu 610041, China; 4 Department of Endocrinology, Affiliated Hospital of Weifang Medical University, Weifang, China; 5 Pediatic Research Institute, Department of Pediatrics, University of Louisville, Louisville, KY, U.S.A.; 6 Wendy L. Novak Diabetes Care Center, University of Louisville, Louisville, KY, U.S.A.

**Keywords:** AMPK, heart failure, substrate metabolism

## Abstract

Heart failure (HF) is a serious disease with high mortality. The incidence of this disease has continued to increase over the past decade. All cardiovascular diseases causing dysfunction of various physiological processes can result in HF. AMP-activated protein kinase (AMPK), an energy sensor, has pleiotropic cardioprotective effects and plays a critical role in the progression of HF. In this review, we highlight that AMPK can not only improve the energy supply in the failing heart by promoting ATP production, but can also regulate several important physiological processes to restore heart function. In addition, we discuss some aspects of some potential clinical drugs which have effects on AMPK activation and may have value in treating HF. More studies, especially clinical trials, should be done to evaluate manipulation of AMPK activation as a potential means of treating HF.

## Introduction

Heart failure (HF) is one of the most common diseases in the United States. Approximately 800000 new cases will be diagnosed every year, causing an enormous economic burden. The direct and indirect costs in 2011 were approximately $320 billion and it is predicted to rise to $918 billion by 2030 [1]. Currently, the therapies of HF attenuating the renin–angiotensin system and the catecholamine response significantly improve the outcomes of HF patients [2]. Even under optimal current therapy, the prognosis of patients suffering from this disease is still poor, with approximately 80% 1-year and 50% 5-year survival rate, which is even lower than the rates of some malignant tumors [1]. Therefore, HF is still a great challenge for clinical physicians and patients. Currently, alternative therapies that could facilitate energy supply and restore the cardiomyocyte homeostasis in the failing heart, are arousing the interests of researchers and physicians.

AMP-activated protein kinase (AMPK) as an energy sensor, regulates multiple physiological processes in the cardiovascular system and could be a potential therapeutic target [3,4]. AMPK has three subunits: α, β, and γ, respectively. Each subunit has multiple isoforms, including α1, α2, β1, β2, γ1, γ2, and γ3, which are encoded by different genes [5]. In the heart, the majority of expressed isoforms are α1/2, β1/2, γ1, and three distinct splice variants of γ2 [6]. The α unit is catalytic, containing a domain of protein kinase. When AMP and ADP bind to γ subunit, they trigger a conformational change in the complex to facilitate the phosphorylation of threonine residue 172 of α subunit. This results in activation of AMPK [7,8]. Other upstream kinases including liver kinase b1 (LKB1) and calcium-calmodulin-dependent kinase kinase 2 (CaMKK2) can also phosphorylate the Thr^172^ activating site to activate AMPK [9]. LKB1 is the main upstream in cardiomyocytes which activates AMPK during ischemia. The insulin-stimulated kinase, Akt can phosphorylate Ser^485^ and Ser^491^ in the α1 and α2 subunits, respectively, which can decrease Thr^172^ phosphorylation of AMPK by LKB1 during ischemia [10].

Much evidence has been published suggesting that activation of AMPK under stress conditions has a protective function in cardiovascular diseases [11–24]. Some reports also showed that AMPK can attenuate the progress of HF [25]. In a rat model of pressure overload-induced cardiac hypertrophy, activity and expression of AMPK are significantly enhanced compared with controls [26]. The cardiac hypertrophy was attenuated by overexpression of adiponectin via activation of AMPK pathway. In mice and humans, the activity of AMPK is also increased in failing hearts [27]. Although, it was demonstrated in one study of HF in mice and humans that the level of activated AMPK was low [28], other studies have found elevated levels during HF [11,26,29,30].

In this context, we will discuss the role of AMPK in HF, especially its protective function involved, in its regulation of metabolism, autophagy, and endoplasmic reticulum stress, and its role in cardiac fibrosis development. Furthermore, we discuss some pharmacological activators of AMPK which have potential for HF treatment.

## AMPK and metabolism in HF

### Metabolism in healthy and failing hearts

The healthy heart is a highly efficient organ. In human, it propels more than 5 l of blood every minute, 7000 l every day, and 2.6 million liters every year [31]. To maintain this work, the heart needs a large energy supply, approximately more than 6 kg ATP per day [32]. In healthy hearts, the main energy comes from fatty acid oxidation, which accounts for 40–60% of ATP production. Fatty acids are transported into the cytosol by fatty acid transporters. Fatty acids bind to coenzyme A (CoA) to form fatty Acyl-CoA, which are then transported into the mitochondria via carnitine palmitoyltransferase I (CPT-1), the limiting step in fatty acid oxidation. Through β-oxidation, fatty acetyl-CoA is converted into acetyl-CoA for ATP production via the tricarboxylic acid (TCA) cycle.

On the other hand, glucose oxidation generates approximately 30% of total cardiac energy production. Glucose metabolism parallels with intracellular glucose concentration. Glucose can enter cardiomyocytes by moving down their concentration gradient via two isoforms of glucose transporters— glucose transporter 1 (GLUT1) and 4 (GLUT4) [33]. Glucose uptake is regulated by the body under different conditions. GLUT1 is responsible for the low level of basal glucose uptake required to sustain respiration in all cells. GLUT4 concentration located in the plasma membrane is regulated as a response to stress. GLUT4 is synthesized in ER, then transported to the Golgi complex where it is modified and budded into the cytosol in a process called sequestration. The protein TUG (tether containing a UBX domain, for GLUT4), mediates the sequestration of GLUT4 storage vesicle (GSV) with one end of TUG attaching to GSVs and the other end anchoring to the cytoskeleton. Under physiological status, most GLUT4 is stored attached to GSVs in the cytosol. However, under stress and insulin stimulation, TUG can then be cleaved to release GLUT4 and the GSVs can fuse with the membrane and transport the GLUT4 to the surface. In addition, translocation of GLUT4 can be regulated by Akt signaling [34–36]. After insulin and/or insulin-like growth factors bind to receptors, insulin receptor substrates (IRS) are phosphorylated and recruited to activate phosphatidylinositide 3-kinase (PI-3K)-Akt pathway. Activated Akt promotes the activity of Rab GTPases by inhibiting AS160/TBC1D4 and TBC1D1, which may facilitate the translocation of GLUT4 to the plasmatic membrane. This process effectively increases glucose uptake [37]. Glucose is transformed to pyruvate in cytosol, which is then transported into the mitochondria and transformed to acetyl-CoA by pyruvate dehydrogenase for further ATP production.

Since glucose and fatty acids are both used as fuel substrates in the heart, the question arises with regard to how the cardiomocytes balance which substrates they will utilize. In 1963, Randle et al. reported the reciprocal relationship between oxidation of fatty acid and glucose, which later became known as the Randle Cycle [38]. When fatty acids increase, β oxidation is enhanced, and glucose oxidation is inhibited. Correspondingly, the increased glucose oxidation can inhibit β oxidation of fatty acids. In contrast, if fatty acid or glucose oxidation is inhibited, oxidation of the other substrate is increased respectively. During pathological conditions, such as hypertrophy, the glucose uptake is enhanced, and this process is considered as a cardioprotective response. Domenighetti et al. [39] demonstrated that deletions of GLUT4 transporters would develop hypertrophy, leading to impaired cardiac systolic function. In a failing heart, the metabolism would be changed (Figure 1). The substrate preference is switched from fatty acid to glucose. However, the production of ATP is markedly decreased. The imbalance between heart energy consumption and ventricular performance is called ‘mechano-energetic uncoupling’. During the early phase of HF, fatty acid oxidation is slightly increased or unchanged. However, glucose utilization is increased. With progression of HF, both fatty acid and glucose oxidation gradually decline, impairing the energy supply to cardiomyocytes. It is unclear whether these changes are adaptive or nonadaptive. Some studies showed that inhibiting mitochondrial CPT-1 and long chain FFA oxidation, consequently increased glycolysis and glucose oxidation, improved the energy supply to cells, and ultimately restored myocardial function and improved symptoms of patients with HF [40–42].

**Figure 1:** Cardiac metabolism in hearts Under normal conditions, cardiomyocytes utilize fatty acids as their major substrate. In the failing heart, the function of mitochondria is impaired. The efficiency of ATP production is dramatically decreased. Cardiomyocytes switch substrate preference to glucose, inducing accumulation of lactate in the failing heart. AMPK regulates multiple related enzymes to promote ATP biosynthesis, ultimately restoring the balance between energy supply and energy demand.

### AMPK helps to restore energy supply and the mitochondrial function

Under pathological conditions, AMPK in hearts is activated as a response to stress. AMPK mediates the transportation of GLUT4 from the cytosol to the membrane, thereby increasing glucose uptake as a cardioprotective and adaptive response of the heart [43]. The translocation of GLUT4 mediated by AMPK refers to phosphorylation of AS160, the Akt substrate protein, which controls many critical steps of cytosol vesicle movement [44]. Moreover, AMPK can inhibit the endocytic cycling of GLUT4 from the membrane, keeping GLUT4 in its active site [45]. Glycolysis is up-regulated by AMPK via phosphorylation of phosphofructokinase 2 (PFK2). AMPK may also inhibit glycogen synthesis and promote the utility of this substrate.

AMPK can also increase fatty acids uptake and oxidation. It increases the translocation of fatty acid transporters CD36 to the membrane, promoting cardiomyocyte uptake of fatty acids. Activated AMPK inhibits acetyl-CoA carboxylase (ACC) by phosphorylation. Consequently, the production of malonyl-CoA is reduced, increasing the activity of CPT-1 [30]. Translocating fatty acids across the mitochondrial membranes by CPT-1 is the rate-limiting step of β-oxidation [46]. Thus, AMPK can increase fatty acid oxidation. All of these effects ultimately increase the ATP production to ameliorate the imbalance between energy supply and energy demand in the failing heart (Figure 1).

Mitochondria are considered to be the ‘powerhouse’, which account for the majority of the ATP production in hearts. They also occupy almost 30% of the volume of matured cardiomyocytes. Apart from oxidative metabolism, mitochondria regulate several physiological signal pathways, supplying cofactors and ligands for biochemical reactions and signal transduction [47,48]. Mitochondrial dysfunction has been widely observed in the failing heart. Therefore, focussing on mitochondria could be a good choice for restoring energy homeostasis in HF. It is reported that the peroxisome proliferator-activated receptor (PPAR) γ coactivator-1α (PGC-1α) is a strong activator in mitochondrial biogenesis in the heart [49]. PGC-1 coactivators regulate the activation of the estrogen-related receptor (ERR) transcription activation. ERRα is an orphan nuclear receptor controlling transcription of genes involved in mitochondrial biogenesis [50]. AMPK can induce mitochondrial biogenesis directly via serine phosphorylation of PGC-1α, or indirectly via the activation of sirtuin 1 (Sirt1), which increases the activity of PGC-1α by deacetylation [51].

Apart from regulation of metabolism in the failing heart, AMPK can also mediate multiple physiological signal pathways (Figure 2). Next, we will discuss the regulatory effects of AMPK on autophagy, ER stress, and cardiac remodeling.

**Figure 2:** AMPK regulates multiple physiological processes to maintain cardiomyocyte homeostasis AMPK activation results in regulation of metabolism, protein transportation, transcription factors, and/or coactivators, kinases, and other enzymes and nonenzymatic proteins. AMPK increases substrate uptake and utilization in cardiomyocytes, enhances mitochondrial biogenesis, and modulates the activity of specific proteins and transcription factors to exert cardioprotective function. Abbreviations: eEF2, eukaryotic elongation factor 2; FAT/CD36, fatty acid translocase; JNK, Jun-amino-terminal kinase; mTOR, mammalian target of rapamycin; ULK1, Unc-51 like kinase 1.

## AMPK and autophagy

Autophagy is a method that the body uses to maintain cellular homeostasis, save energy, and appropriately distribute energy utility. Autophagy can degrade unwanted protein. During the process, the cytosolic cargo is delivered to the lysosome for degradation. The products of degradation are transported back to cytosol for biosynthesis or energy production. Autophagy can also restore mitochondrial function and clear excessively produced reactive oxygen species (ROS) as an adaptive and defensive mechanism [52]. Autophagy plays an essential role in cardiovascular injuries, by maintaining cellular function under basal conditions as well as in response to stress [53–56]. During cardiac hypertrophy, appropriate autophagy can restore cardiac structure and function. Several studies reported that autophagy is involved in the development of cardiac hypertrophy, and the remodeling during hypertrophy deteriorates when autophagy is inhibited in hearts [57,58]. The mammalian target of rapamycin (mTOR) is an energy sensor involved in balancing nutrient status and cell growth. Under sufficient nutrient conditions, mTOR promotes cell growth partially by inhibiting autophagy. However under nutrient-insufficient conditions, mTOR is inactivated and autophagy is enhanced [52]. Rapamycin, as an inhibitor of mTOR complex 1 (mTORC1), promotes autophagy, thus increasing cell survival and cardioprotection [59]. Li et al. [60] demonstrated that AMPK protects the heart in stress of pressure overload-induced hypertrophy by enhancing autophagy via mTORC1 inactivation. AMPK phosphorylates tuberous sclerosis complex 2 (TSC2), the negative regulator of mTORC1, to inhibit mTORC1 activity and its downstream target p70S6K and promote autophagy [61]. This signaling pathway is essential to maintain heart function under stress conditions [62]. Apart from indirectly increasing autophagy via inhibiting mTORC1, AMPK can also directly induce autophagy by phosphorylating the Unc-51 like kinase 1 (ULK1) kinase complex, which is the mammalian homolog of yeast Atg1 [63].

Intriguingly, appropriate autophagy maintains cardiac homeostasis, however, excessively activated autophagy may result in cell death and deterioration of heart hypertrophy. Liu et al. [64,65] reported that suppressing the CaMKKβ-AMPK-mTOR pathway to down-regulate autophagy has cardioprotection in prolonged stimulation-induced cardiac hypertrophy. Another study showed that increased autophagy in the heart led to impaired cardiac function, suggesting that prolonged activation of autophagy might be harmful to the heart [66]. In the future, further research into the function of autophagy and its role in HF may lead to new therapies based on the modulation of autophagy.

## AMPK and ER stress

The ER is an organelle modulating protein biosynthesis and appropriate folding, calcium homeostasis, lipid biosynthesis, and cell apoptosis [67]. Multiple stimuli, such as hypoxia, ROS, elevated protein synthesis, and calcium overload, can cause ER dysfunction.

During HF, ER stress also plays a role. There is evidence supporting that apoptosis of cardiomyocytes induced by ER stress contributes to cell loss in HF [68,69]. Normal functioning ER can help the protein fold properly. During HF, accumulation of unfolded protein induces ER stress. Progressive ER stress can induce apoptosis of cardiomyocytes [70]. Okada et al. [71] investigated ER stress in pressure-overload induced hearts. They found that HF can induce prolonged ER stress, up-regulating the expression of C/EBP-homologous protein (CHOP), thereby resulting in cardiomyocyte apoptosis during the progression from hypertrophy to HF.

Several papers demonstrated that AMPK activation can influence ER stress, however, the exact mechanism is still unknown. Terai et al. [72] found that activating AMPK by AICAR attenuated ER stress in neonatal rat cardiomyocytes, with reduction in CHOP expression and cleaved caspase 12. The mechanism of this process is probably through activated AMPK attenuating protein synthesis via eukaryotic elongation factor 2a (eEF2a) inactivation [72]. Furthermore, Zhuo et al. [73] demonstrated that in a rat model of HF induced by prolonged isoproterenol stimulation, aberrant ER stress is induced with heart dysfunction, BNP elevation, and cardiomyocyte apoptosis—all of which can be inhibited by AMPK activation. Lu et al. [74] reported that ER stress-related markers, such as GRP78, CHOP, and caspase-12 were overexpressed in the rat HF model induced by abdominal aortic constriction. As a novel member of the calcitonin/calcitonin gene-related peptide family, Intermedin was discovered to improve heart function, reduce ER stress, and ameliorate cardiomyocyte apoptosis via an AMPK-dependent pathway [74]. Park et al. [75] demonstrated that AMPK possibly mediated ER stress through mTOR pathway. AMPK can inhibit mTOR activity, resulting in attenuation of new protein synthesis, reducing the accumulation of unfolded proteins, and thereby reducing ER stress [75]. However, the detailed mechanisms of how AMPK mediates ER stress to protect the heart from HF need to be further elucidated.

## AMPK and cardiac remodeling

The remodeling process of the heart can be induced by stresses such as ischemia and pressure overload, eventually leading to hypertrophy or dilation of ventricles. During this process, not only cardiomyocytes, but also endothelial cells, immune cells, and fibroblasts are involved. Furthermore, several different hormones play roles in this process, such as angiotensin, catecholamine, and endothelins, and some inflammatory cytokines including IL1-b, IL-6, TGF-β, and TNF-α. Myocardial fibrosis is a result of ECM remodeling, with increased myocardial stiffness and impaired pumping capacity contributing to HF. Myocardial fibrosis can be categorized as two types: reactive interstitial fibrosis and reparative fibrosis [76]. Reactive interstitial fibrosis triggered by stress is a defensive response without cell death, but associated with ECM deposition. However, reparative fibrosis involves cardiomyocyte necrosis and the formation of collagen scar tissue. Excessive ECM deposition and formation of scar tissue causes stiffness of myocardium and reduction in ventricular compliance, leading to diastolic dysfunction. The progression of cardiac fibrosis induces ventricular dilation and impairment of systolic function, and ultimately HF.

According to a few studies, AMPK plays a protective role in the process of cardiac fibrosis. TGF-β is considered a potent profibrogenic cytokine in the pathogenesis of cardiac fibrosis [77]. It regulates cell proliferation, inflammation, and deposition of ECM. It is also the critical factor involved in activation and/or differentiation of cardiac fibroblasts [78]. Of the three isoforms of TGF-β, TGF-β1 is dominant in hearts. Smad proteins (mainly Smad2/3) are downstream in the TGF-β pathway, which translocates into the nucleus promoting the transcription of specific genes [79]. Xiao et al. showed that the TGF-β/Smad3 signaling pathway plays a role in pressure overload-induced cardiac fibrosis [80]. Additionally, TGF-β1 can also activate some signaling pathways independent from Smad, including extracellular signal-regulated kinase (ERK), c-Jun N-terminal kinase (JNK), and p38 mitogen-activated protein kinase (p38 MAPK) [80]. The up-regulation of these pathways is related to myofibroblast activation. However, AMPK activation can regulate TGF-β transcription by suppressing the expression of hepatocyte nuclear factor (HNF-4) in cardiac fibroblasts [81]. ERK is critical in regulating growth and proliferation of cardiac fibroblasts. Du et al. [82] reported that the activation of AMPK inhibits the activity of cardiac fibroblasts by inhibiting ERK. Chen et al. [83] reported that AMPK modulated JNK-NF-κB signaling cascade. The inhibition of JNK and NF-κB via AMPK activation can attenuate the inflammation and cell death to protect cardiomyocytes [83].

ROS are also related to the progression of cardiac fibrosis, and ROS scavenger treatments have cardioprotective function [84]. Several studies demonstrated that reducing ROS levels via AMPK-dependent pathway can attenuate cardiac fibrosis [85,86].

## Drugs modulating AMPK which may have clinical value in treating HF

Few studies demonstrated whether AMPK activation in HF is temporary or constant. However, AMPK activation is shown to have cardioprotective function not only in metabolism but also in other aspects of physiological function. It is reasonable that pharmacological activation of AMPK could be a treatment strategy to improve cardiac energy supply and mechanical function in patients with HF. Some drugs were reported to have effects on activating AMPK, such as metformin, statin, trimetezidine, and resveratrol, and may have potential to be used clinically for therapy of HF in the future [87].

### Metformin

Metformin is commonly used clinically for treatment of diabetes. But more and more researches, both *in vitro* and *in vivo* experiments, have demonstrated that it can activate AMPK, with either direct or indirect mechanisms [88,89]. Interestingly, in both acute and chronic treatment of diabetes, administration of metformin failed to increase intracellular total AMPK level, but rather simply increased the activity of AMPK by enhancing its phosphorylation [90,91]. The direct mechanism of metformin activating AMPK might involve the binding of AMPK subunits, increasing the assembly of heterotrimeric complexes, which is more easily accessed by upstream kinases [92,93]. In addition to the direct pathway, metformin is also able to activate AMPK indirectly by altering the AMP or ADP/ATP ratio. The details may be complicated, but at least two ways are clear. One is that metformin can inhibit the activity of AMP-deaminase. The other is that it can inhibit the respiratory chain by inhibiting mitochondrial complex 1 [94]. Both of them can result in increase in AMP or ADP/ATP ratio and then induce the activation of AMPK.

Some studies show that metformin alleviates cardiac hypertrophy in chronic pressure overload mice through an AMPK pathway. Metformin has also been shown to reduce cardiac fibrosis and inhibit collagen synthesis in hypertrophied hearts [95]. In oxidative stress-induced cardiomyocyte hypertrophy, metformin protects the CM partially through the AMPK-eNOS pathway. In a rat model of isoproterenol-induced cardiac hypertrophy, metformin per oral can prevent myocardial injury and fibrosis, dose-dependently [96]. In a dog model of tachycardia-induced HF, metformin promoted phosphorylation of both AMPK and endothelial nitric oxide synthase, increased plasma nitric oxide levels, and improved insulin resistance, resulting in reduction in CM apoptosis and improvement of cardiac function [97]. In a mice model of press overload induced HF, metformin improved left ventricular systolic function and ventricular remodeling [98].

### Trimetazidine

Trimetazidine (1-[2,3,4-trimethoxibenzyl]- piperazine) (TMZ), can selectively inhibit long-chain 3-ketoacyl-co-enzyme A (CoA) thiolase (3-KAT), which is the key enzyme involved in fatty acids β-oxidation, shifting substrate metabolism in hearts from fatty acids oxidation to glucose oxidation [99].

Saeedi et al. [100] reported that in hypertrophied rat hearts, TMZ stimulated glucose oxidation and reduced proton production, thereby improving cardiac function. Several randomized clinical trials (RCTs) have demonstrated that TMZ can improve patients’ New York Heart Association (NYHA) Functional Classification, heart function, exercise tolerance, and quality of life [101–103]. In the up to 6 months follow-up study, Brottier et al. [104] reported that 20 patients with severe ischemic cardiomyopathy receiving TMZ treatment had an improvement in NYHA class and heart function. Some other studies also showed that, after TMZ treatment in patients with HF, cardiac function and remodeling was improved along with a reduction in inflammatory response, B-type natriuretic peptides, and cardiac troponin levels [101,105].

Although most studies have investigated the effects of TMZ in patients with HF caused by ischemic cardiomyopathy, a few studies have demonstrated the effectiveness of continuous TMZ treatment in HF caused by nonischemic etiology [106–108]. In 19 patients with HF induced by idiopathic dilated cardiomyopathy, administration of TMZ can improve EF (the ejection fraction) of hearts and whole-body insulin sensitivity [106]. Zhao et al. [107] investigated patients with diabetes and idiopathic dilated cardiomyopathy, receiving TMZ (20 mg, t.i.d) for 2 months, showing that TMZ treatment improved cardiac function and physical tolerance, and reduced the inflammatory response.

Suppression of fatty acid oxidation by TMZ can decrease NADH/NAD^+^ ratio, induce enhancement of PDH activity, and increase glucose and pyruvate oxidation. Therefore, TMZ treatment can shift substrate metabolism in the heart. Besides, Liu et al. [109] reported that TMZ can increase the activity of AMPK by influencing the ATP level in cardiomyocytes. Therefore, the mechanism in which TMZ protects the heart from HF may function through an AMPK pathway. However, the details are still not clear.

### Statins

Statins, are inhibitors of the hydroxymethylglutaryl-CoA (HMG-CoA) reductase enzyme. By inhibiting a key step in the sterol biosynthesis, statins are important cholesterol lowering medications and have amazing effects on prevention of cardiovascular disease [110]. The effects beyond cholesterol control effects of statins are called pleiotropic effects. Many studies have demonstrated that administration of statin protects hearts from heart remodeling. Treatment with atorvastatin for 4 weeks attenuates heart dysfunction, fibrosis, and hypertrophy after MI in rats, and also lowers expression levels of inflammatory cytokines such as TLR4, IL-1, and NF-kB [84]. The efficacy of statin treatment in improving prognosis of cardiovascular disease has been proven in different clinical trials [111–113]. These cardioprotective functions, especially resistance of cardiac fibrosis, may be mediated by AMPK activation [114,115]. In the studies of Chen et al. [116–118], Izumi et al. [116–118], and Sun et al. [116–118], it was reported that statins can activate eNOS signaling pathway via AMPK, to control NO bioavailability and maintain cardiovascular homeostasis. The detailed mechanisms by which statin can activate AMPK still needs further review, however, multiple studies have demonstrated that statins may activate AMPK by altering the AMP/ATP ratio or increasing ROS-dependent PKCξ activity [119,120].

### Resveratrol

Resveratrol (3,4′,5-*trans*-trihydroxystilbene) is a natural antioxidant found in numerous plant species, including red grapes, berries, and peanuts [121]. More and more studies have supported the beneficial effect of resveratrol in HF. Chan et al. [122] demonstrated that resveratrol is able to inhibit cardiomyocyte hypertrophy through an AMPK-dependent pathway. This process is dependent on the presence of AMPK upstream kinase, LKB1. Zordoky et al. [121] reported that resveratrol inhibits cardiac hypertrophy by reducing oxidative stress through an AMPK-dependent mechanism. In contrast, Wang et al. [123] found that resveratrol attenuated HF in a rat model by inactivating AMPK and thereby inhibiting autophagy. However, other studies support that resveratrol improves cardiac function in HF by activating Sirt1 and up-regulating AMPK [124]. The mechanism by which resveratrol activates AMPK is complicated, but at least two possible mechanisms were recently discovered [125]. One is that resveratrol delivered at a high concentration (50–100 μM) can activate AMPK by increasing AMP/ATP ratio. On the other hand, resveratrol might activate AMPK via Sirt1-LKB1. Wang et al. [126] showed that Sirt1 deacetylases LKB1 to facilitate LKB1–AMPK association, and thereby increase AMPK activity. Interestingly, these activation mechanisms vary amongst different cell types, with some cell types failing to activate AMPK through resveratrol treatment.

Although some of these drugs are already used clinically, they are not specific for HFfailure currently. On the other hand, a number of animal studies have demonstrated that these drugs may be used for the treatment of cardiovascular disease. However, the bioavailability, pharmacodynamics or side effects of these drugs may block their utility in clinical trials or practices. As an alternative strategy, some new analogs or drug-delivery systems, may facilitate the administration of these drugs as new clinical therapies for HF [127].

## Conclusion

HF is the result of a variety of pathophysiological processes originating from dysfunctional metabolism, mitochondrial function, inflammation, and apoptosis. As an energy regulator, AMPK not only improves energy supply to increase heart function, but also improves HF and heart function by mediating various intracellular physiological functions, delaying myocardial fibrosis, and reducing heart damage. Some drugs already used in clinical medicine, such as metformin, statin, TMZ, resveratrol etc., have the function of activating AMPK, and may be used as an alternative drug for treatment of HF in the future.

## Abbreviations

AICAR: 5-aminoimidazole-4-carboxamide ribonucleotide
AMPK: AMP-activated protein kinase
BNP: B-type natriuretic peptide
C/EBP: CCAAT-enhancer-binding protein
CHOP: C/EBP-homologous protein
CM: cardiomyocyte
CoA: coenzyme A
CPT-1: carnitine palmitoyltransferase I
ECM: extracellular matrix
eNOS: endothelial nitric oxide synthase
ER: endoplasmic reticulum
ERK: extracellular signal-regulated kinase
ERR: estrogen-related receptor
GLUT: glucose transporter
GRP78: 78-kDa glucose regulated protein
GSV: GLUT4 storage vesicle
HF: heart failure
IL: interleukin
JNK: c-Jun N-terminal kinase
LKB1: liver kinase b1
MI: myocardial infarction
mTOR: mammalian target of rapamycin
mTORC1: mTOR complex 1
NF-κB: nuclear factor kappa-light-chain-enhancer of activated B cells
NYHA: New York Heart Association
PDH: pyruvate dehydrogenase
PGC-1α: peroxisome proliferator-activated receptor γ coactivator-1α
PKC: protein kinase C
ROS: reactive oxygen species
Sirt1: sirtuin 1
Smads: the homologies of the *Caenorhabditis elegans* SMA and Drosophila MAD family of genes.
TGF-β: transforming growth factor beta
t.i.d: ter in die (three times a day)
TLR4: Toll-like receptor 4
TMZ: trimetazidine
TNF-α: tumor necrosis factor alpha
TUG: tether containing a UBX domain, for GLUT4
